# Pentoxifylline as an adjunctive in treatment of negative symptoms in chronic schizophrenia: A double‐blind, randomized, placebo‐controlled trial

This article has been retracted.

**DOI:** 10.1111/cns.14010

**Published:** 2022-11-07

**Authors:** Mahmoud S. Abdallah, Esraa M. Mosalam, Ahmed Hassan, Ahmed N. Ramadan, Hend Omara‐Reda, Abdel‐Aziz A. Zidan, Waad A. Samman, Eman I. El‐berri

**Affiliations:** ^1^ Department of Clinical Pharmacy, Faculty of Pharmacy University of Sadat City Sadat City Egypt; ^2^ Department of Biochemistry, Faculty of Pharmacy Menoufia University Shebeen El‐Kom Egypt; ^3^ Department of Neuropsychiatry, Faculty of Medicine Menoufia University Shebeen El‐Kom Egypt; ^4^ Zoology Department, Faculty of Science Damanhour University Damanhour Egypt; ^5^ Department of Pharmacology and Toxicology, College of Pharmacy Taibah University Medina Saudi Arabia; ^6^ Clinical Pharmacy Department, Faculty of Pharmacy Tanta University Tanta Egypt

**Keywords:** inflammatory cytokines, negative symptoms, PANSS, pentoxifylline, phosphodiesterase inhibitor, schizophrenia

## Abstract

**Aim:**

The aim of this study was to explore the effectiveness and safety of pentoxifylline as an adjuvant to risperidone in mitigating the negative symptoms in patients with chronic schizophrenia.

**Methods:**

In this randomized, placebo‐controlled study, eighty outpatients with chronic schizophrenia were given risperidone for 8 weeks along with either pentoxifylline or a placebo. The positive and negative syndrome scale (PANSS) was used to assess patients at the start of the trial, as well as at 2, 4, 6, and 8 weeks. Pre‐ and posttreatment serum levels of cAMP, TNF‐α‐, and IL‐6 were measured.

**Results:**

The pentoxifylline group revealed a significant effect for time‐treatment interaction on PANSS‐negative subscale scores (*p* < 0.001), PANSS general psychopathology subscale scores (*p* < 0.001), and PANSS total scores (*p* < 0.001), but not on PANSS‐positive subscale scores (*p* = 0.169). Additionally, when compared to the placebo group, the pentoxifylline group demonstrated a statistically significant increase in cAMP serum level and a statistically significant decrease in TNF‐α and IL‐6 serum levels.

**Conclusion:**

Pentoxifylline adjunctive therapy with risperidone for 8 weeks was found to be promising in mitigating the negative symptoms in patients with chronic schizophrenia. Trial registration number: NCT04094207.

## Graphical abstract

Phosphodiesterases and inflammation play a role in the pathophysiology of schizophrenia negative symptoms. Treatment with the PDE inhibitor pentoxifylline improve the expression of cAMP and decreases the expression of inflammatory cytokines including TNF‐α and IL‐6. Upregulation of cAMP/PKA signaling triggers the synthesis of dopamine at dopaminergic synapse, blocks the dopamine D2‐receptor, and activates dopamine D1‐receptor in striatonigral neurons. Pentoxifylline adjunctive therapy with risperidone for 8‐weeks demonstrated a favorable efficacy and safety profile in improving the negative symptoms in patients with chronic schizophrenia.

## 1 INTRODUCTION

Schizophrenia is a chronic psychiatric disorder that contributes significantly to the burden of mental disease worldwide.^1^ The main challenge that faced many researchers is the negative symptoms, which are responsible for functional impairment and poor outcomes.^2^ Negative symptoms include reduction or absence of motivational and interest‐related behaviors as avolition, anhedonia, social withdrawal, or expression such as alogia and affective flattening.^3^ About 30% of patients with schizophrenia are resistant to the available treatment.^4^ Antipsychotics have no satisfactory effect on alleviating the negative symptoms; besides, the Food and Drug Administration did not approve any drugs concerning these symptoms.^5^ However, evidence showing the effectiveness of the antipsychotic cariprazine in the management of the negative symptoms in large‐scale clinical trial.^6^ Moreover, adjunctive antidepressants have shown modest efficacy in alleviating negative symptoms (e.g., duloxetine).^7^ Other medications that have been tried in conjunction with antipsychotics to alleviate negative symptoms with potential effectiveness include minocycline,^8^ dopamine agonists (e.g., selegiline, modafinil), cholinergics (e.g., galantamine, donepezil),^3^ antidiabetics (e.g., pioglitazone),^9^ and anti‐inflammatory (e.g., celecoxib).^10^, ^11^

Several attempts have been made to define the distinctive mechanisms responsible for these negative symptoms to introduce new therapeutic agents that could target those mechanisms.^7^, ^12^ Several studies' findings have suggested that inflammatory cytokines involving tumor necrosis factor‐alpha (TNF‐α) and interleukins, as well as neurobiological pathways such as the serotonergic, dopaminergic, and glutamatergic pathways, may have a role in the emergence of these symptoms.^4^, ^13^, ^14^ Previous studies have explained the role of phosphodiesterases (PDEs) in schizophrenia pathogenesis. Inhibition of PDEs decreases dopamine D2‐mediated signaling while enhancing dopamine D1‐dependent signaling, suggesting that it could be used to treat dopamine D1‐dependent signaling and reward processing impairments in individuals with negative symptoms.^15^, ^16^ Therefore, PDEs could be a promising therapeutic target.^17^ PDEs are enzymes that hydrolyze cyclic nucleotides and hence play an important role in modulating intracellular levels of both cyclic adenosine monophosphate (cAMP) and cyclic guanosine monophosphate (cGMP).^18^ Elevated cAMP can induce the synthesis of different neurotransmitters such as glutamate and dopamine.^19^, ^20^ Inside the cells, the effect of dopamine on neurons is basically influenced by cAMP‐activated pathways.^21^ Furthermore, it has been suggested that cGMP modulation could be a strategy for dealing with negative symptoms.^22^

Studies over the past two decades have provided important data about the effects of inflammatory cytokines, involving TNF‐α, interleukin‐1beta (IL‐1β), and IL‐6, on the basal ganglia, which contributes to the pathogenesis of all neuropsychiatric diseases including negative symptoms and motivational deficits.^4^, ^23^ Moreover, many psychotropic medications have “anti‐inflammatory” properties, and as a result, numerous “anti‐inflammatory” agents have been studied for their potential therapeutic effects in various psychiatric disorders.^24^ Changes in peripheral inflammatory biomarkers have been identified in patients with schizophrenia with acute progression of the symptoms and in chronic patients where negative symptoms are more remarkable.^25^ Additionally, inflammation could affect dopaminergic and glutamatergic signaling by decreasing dopamine availability and release, as well as decreasing concentrations of tetrahydrobiopterin, a cofactor required for dopamine synthesis.^26^ Furthermore, proinflammatory cytokines reduce glutamate transporter expression on the astrocyte cell surface and increase glutamate release.^27^ Evidence suggests that dopamine and glutamate have downstream effects on connectivity in brain circuitry in schizophrenia patients, including disrupted resting state networks.^4^

Pentoxifylline is a methylated xanthine derivative and works as a phosphodiesterase inhibitor that is commonly used for the management of claudication symptoms by inhibition thrombocytes aggregation, boosting erythrocyte flexibility or deformity, and decrease blood viscosity.^28^, ^29^ Off‐label use of pentoxifylline includes venous ulcers and severe alcoholic hepatitis management. The most common side effects of pentoxifylline are nausea and vomiting, followed by abdominal discomfort, bloating, diarrhea, dizziness, headache, and flushing.^30^ The rationale for pentoxifylline usage in schizophrenia is that it competitively inhibits 5′‐nucleotidase and PDE4 and PDE5, resulting in enhanced intracellular cAMP, protein kinase A (PKA) activation, and suppression of interleukins and TNF‐α production, which ultimately reduce inflammation.^31^, ^32^ Moreover, it was reported that pentoxifylline could be safe and effective adjuvant in some neuropsychiatric disorders including depression^33^ and autism.^31^ These properties suggest that it could be a promising adjuvant therapy in schizophrenia patients. As a result, the aim of this randomized, double‐blind, placebo‐controlled trial was to explore the effectiveness and safety of pentoxifylline as an adjuvant to risperidone in mitigating the negative symptoms in patients with chronic schizophrenia.

## 2 METHODS

### 2.1 Study design

This study was a prospective, parallel‐group, randomized, double‐blind, 8‐week trial. The Menoufia University Faculty of Medicine's ethical committee granted approval for this study (4/2021NEUR1), and it was carried out in accordance with the Declaration of Helsinki and its subsequent amendments. The study was registered at ClinicalTrials.gov (NCT04094207). The recruited patients or their legal representatives signed printed informed consent forms. The trial's open‐ended withdrawal policy was disclosed to the participants.

### 2.2 Participants

From September 2019 to January 2022, patients between the ages of 20 and 40 were recruited from the neuropsychiatric department of Menoufia University Hospital. Patients with a confirmed diagnosis of schizophrenia using a structured interview conducted in accordance the Diagnostic and Statistical Manual of Mental Disorders, 4th Edition, Text Revision,^34^ a minimum 2‐year history of schizophrenia, and a serum C‐Reactive Protein (CRP) level ≥5 mg/dl, which was determined in a clinical laboratory prior to enrollment as a sign of low‐grade inflammation, were eligible.^35^ Patients must be able to give informed consent, be willing to take medication orally, be stable on risperidone for at least 8 weeks, be clinically stable as determined by the treating doctor, and not have needed an increase in antipsychotic medication over the past 4 weeks.

Exclusion criteria included abusing alcohol or other drugs, having intellectual disability, having undergone electroconvulsive therapy within the previous 12 weeks, having any other mental disorders, scoring ≥4 on the depression item of the positive and negative syndrome scale (PANSS)^36^ or scoring ≥14 on the 17‐item Hamilton depression rating scale (HDRS).^37^ Furthermore, pentoxifylline hypersensitivity, any life‐threatening illness or neurological disorder, major extrapyramidal symptoms, abnormal bleeding history, pregnant or nursing women, or females intending pregnancy were all prohibited. The discontinuing criteria were the patient's appeal, the decision of the responsible medical investigator (e.g., adverse effect, inadequate compliance), and gestation.

### 2.3 Sample size

With an effect size (Cohen's *d*) ≥0.75, a sample size of 40 patients in each group would have 80% power to identify any potential benefits for pentoxifylline on the PANSS total scores when compared to placebo with the following assumptions: a mean difference of three between the two groups' PANSS total scores, a standard deviation (SD) of 4, an alpha error of 0.05, beta error of 0.2, and 15% attrition rate. It is worth noting that the power of repeated measures analyses is significantly higher.

### 2.4 Randomization and blinding

Randomization was performed by impartial person using electronic random number generator. (Assignment ratio was 1:1, blocks of two). Blinding of the assignment was achieved by using serially numbered, solid, and stapled wrappers. Placebo tablets were manufactured in Zeta Pharma Company, and they were indistinguishable from pentoxifylline tablets in their appearance. The assignment was concealed from the participant, the doctor who referred the patient, the healthcare provider, the statistician, and the evaluator.

### 2.5 Intervention

Pentoxifylline 400 mg SR tablets twice day, or a placebo, were given to participants for 8 weeks. Pentoxifylline dose selection was based on our previous study^33^ to minimize the side effects and enhance patient compliance and adherence. Risperidone was administered to all patients up to 6 mg/day. The drugs were given out by the pharmacist, and the pills that had been resumed were tested for adherence.

### 2.6 Outcomes

The PANSS validated 30‐item rating scale, which comprises positive (seven items), negative (seven items), psychopathological symptoms in general (16 items), and PANSS total scores, was used to assess the drug efficacy and severity of symptoms in patients with schizophrenia.^36^ The PANSS evaluation was based on a structured clinical interview at the beginning of the trial, as well as at weeks 2, 4, 6, and 8. The primary outcome measure in both groups was the change in PANSS negative subscale scores from baseline to week 8. The secondary outcome compared changes in PANSS total and subscale scores between groups from baseline to each time point. Furthermore, HDRS was measured at the beginning and at week 8 to evaluate the depressive symptoms using 17‐rating item scale.^37^ Extrapyramidal Symptoms Rating Scale (ESRS; part one: parkinsonism, dystonia, dyskinesia)^38^ was used to evaluate extrapyramidal symptoms at each visit. Other outcome included cAMP, TNF‐α, and IL‐6 serum levels for biological evaluation of the medications after therapy.

### 2.7 Safety

Patients were advised to notify the study team if they experienced any unusual symptoms during the trial. At each appointment, adverse effects (AEs) were meticulously recorded using a checklist. Physical examinations were also performed, and the participants' vital signs and body weight were listed during the screening session. Patients or their representatives were called once a week to assess their adherence to the medications.

### 2.8 Measurements

Fasting morning blood samples (10 a.m.) were collected at the same time for all patients in vacutainers. The samples were then centrifuged at 4500 *g* for 15 min to separate the serum, which was transferred to eppendorf tubes and stored at −80°C deep freezer until analysis. Specific commercial ELISA kits (MyBioSource, Inc.) were used to determine cAMP, TNF‐α, and IL‐6 serum levels according to supplier's instructions with catalogue number MBS163681, MBS267654, and MBS261259, respectively. The intra‐ and interassay coefficients of variation for cAMP were 8.4% and 8.2%, for TNF‐α were 8.6% and 8%, and for IL‐6 were 7.8% and 7.2%, respectively.

### 2.9 Statistical analysis

Data analysis was done using IBM® SPSS® Statistics version 22 software (USA). Shapiro–Wilk and Kolmogorov–Smirnov tests were used to examine the normal distribution of continuous variables. Student's *t* test was used to compare independent samples with normal distribution of continuous variables, and the Wilcoxon rank sum test was utilized if the normality assumptions of the *t* test were not met. Continuous variables with normal distribution were reported as mean ± SD. The chi‐square test or Fisher's exact test as appropriate used for the frequencies of categorical data. PANSS, HDRS, and ESRS scores were compared using a general linear model repeated measure. If Mauchly's test of sphericity proved significant, the Greenhouse–Geisser correction for degrees of freedom was used. For multiple tests, a Bonferroni correction was used to control type 1 error. Multiple linear regression analysis was used when PANSS‐negative symptoms showed substantial reductions, with changes in PANSS positive and general scores, HDRS, and ESRS scores, as well as the treatment groups, as predictors. The Pearson's correlation was used to assess the relationship between the variables. GraphPad Prism 6.01 software is used for Graphs creation.

## 3 RESULTS

According to the inclusion and exclusion criteria, 116 patients were assessed for their eligibility. Eighty outpatients were randomized to receive either pentoxifylline or placebo (*n* = 40 for each). After a week, six participants withdrew from the trial. Seventy‐four patients (37 in each group) completed the trial, and they were considered in the ensuing analyses (Figure 1). When compared between the two groups, baseline participant characteristics, PANSS total and subscale scores, HDRS score, and ESRS score were not substantially different (Table 1). At the beginning, all patients' HDRS scores were ≤9.

**FIGURE 1:** Flow chart of the study participants

**TABLE 1:** Participants' demographics and baseline characteristics

	Placebo group (*n* = 40)	Pentoxifylline group (*n* = 40)	Statistical value
Age (years)	31.6 ± 4.3	32.73 ± 8.38	*p* = 0.391
Gender			
Male	21 (52.5%)	19 (47.5%)	*p* = 0.823
Female	19 (47.5%)	21 (52.5%)	*p* = 0.823
Smoking	17 (42.5%)	19 (47.5%)	*p* = 0.822
Weight (kg)	69.9 ± 6.4	70.38 ± 7.19	*p* = 0.759
Height (cm)	169.25 ± 6.51	170.18 ± 7.94	*p* = 0.57
BMI (kg/m^2^)	24.41 ± 1.92	24.29 ± 1.88	*p* = 0.793
Marital status			
Single	10 (25%)	12 (30%)	*p* = 0.921
Married	15 (37.5%)	14 (35%)	*p* = 0.921
Divorced	15 (37.5%)	14 (35%)	*p* = 0.921
Education level			
Illiterate	2 (5%)	3 (7.5%)	*p* = 0.921
Primary school	16 (40%)	15 (37.5%)	*p* = 0.921
High school diploma	12 (30%)	10 (25%)	*p* = 0.921
University degree	10 (25%)	12 (30%)	*p* = 0.921
Type of schizophrenia			
Paranoid	32 (80%)	30 (75%)	*p* = 0.924
Residual	4 (10%)	6 (15%)	*p* = 0.924
Disorganized	4 (10%)	4 (10%)	*p* = 0.924
Baseline scores, mean ± SD			
PANSS total score	70.6 ± 6.59	72.65 ± 7.41	*p* = 0.444
PANSS general subscale score	35.23 ± 3.81	35.35 ± 4.12	*p* = 0.888
PANSS negative subscale score	17.43 ± 1.99	17.93 ± 2.14	*p* = 0.282
PANSS positive subscale score	18.33 ± 1.85	18.88 ± 2.11	*p* = 0.219
PANSS cognitive factor	7.025 ± 0.77	7.275 ± 0.88	*p* = 0.179
HDRS score	7.55 ± 0.85	7.35 ± 0.95	*p* = 0.323
ESRS score	1.74 ± 0.42	1.73 ± 0.45	*p* = 0.566
Time from first psychosis (months)	27.48 ± 1.5	27.82 ± 1.36	*p* = 0.277
CRP (mg/dl)	6.27 ± 1.03	6.63 ± 1.27	*p* = 0.168

*Note*: Data presented as mean ± SD. Abbreviations: BMI, body mass index; CRP, C‐Reactive Protein; ESRS, Extrapyramidal Symptoms Rating Scale; HDRS, Hamilton Depression Rating Scale score; PANSS, Positive and negative syndrome scale score.

### 3.1 Outcomes

#### 3.1.1 PANSS‐negative symptoms

No significant differences were found between the two groups' baseline PANSS‐negative subscale scores (*p* = 0.282). The PANSS‐negative subscale scores significantly changed as a result of the time‐treatment interaction in the general linear model repeated measures [*F* (2.665, 191.89) = 84.58, *p* < 0.001, η^2^ = 0.54] (Figure 2A). When comparing the two groups' PANSS‐negative subscale scores, the pentoxifylline group displayed noticeably greater decreases from week four to week eight (Table 2). Moreover, the treated group was also a significant predictor of changes in negative symptoms in this trial, according to our results from multiple linear regression (standardized β = 0.701, β = 2.757, *t* = 8.339, *p* < 0.001).

**FIGURE 2:** The two therapies' effects on the Positive and Negative Syndrome Scale (PANSS). Data presented as means ± SD: (A) Negative, (B) Positive, (C) General psychopathology, and (D) Total scores. NS, non‐significant

**TABLE 2:** Baseline‐to‐endpoint decline in PANSS scores

Outcome	Placebo group (*n* = 37) mean ± SD	Pentoxifylline group (*n* = 37) mean ± SD	Statistical value	Cohen's *d*
PANSS‐negative subscale score				
Week 2	0.68 ± 0.47	0.7 ± 0.46	*p* = 0.805	0.058
Week 4	1.7 ± 0.46	3.0 ± 0.71	*p* < 0.0001	2.8
Week 6	1.95 ± 0.23	4.46 ± 1.26	*p* < 0.0001	2.77
Week 8	2.84 ± 0.37	5.85 ± 1.59	*p* < 0.0001	2.6
PANSS‐positive subscale score				
Week 2	1.57 ± 0.65	1.59 ± 0.6	*p* = 0.853	0.043
Week 4	2.81 ± 0.4	2.78 ± 0.71	*p* = 0.841	0.047
Week 6	3.49 ± 0.56	3.65 ± 0.89	*p* = 0.351	0.218
Week 8	4.49 ± 0.73	4.65 ± 1.23	*p* = 0.493	0.16
PANSS general subscale score				
Week 2	1.41 ± 0.5	1.32 ± 0.75	*p* = 0.585	0.128
Week 4	2.49 ± 0.61	2.7 ± 1.02	*p* = 0.273	0.257
Week 6	3.84 ± 0.37	5.03 ± 0.87	*p* < 0.001	1.78
Week 8	4.68 ± 0.49	6.08 ± 1.06	*p* < 0.001	1.706
PANSS total score				
Week 2	3.77 ± 1.2	3.62 ± 1.34	*p* = 0.921	0.023
Week 4	7.89 ± 1.9	8.49 ± 1.73	*p* = 0.11	0.33
Week 6	9.27 ± 0.73	13.14 ± 1.85	*p* < 0.001	2.71
Week 8	12.0 ± 1.22	16.84 ± 3.52	*p* < 0.001	2.12

Abbreviation: PANSS, Positive and negative syndrome scale score.

#### 3.1.2 PANSS‐positive symptoms

When comparing the two groups, the baseline PANSS‐positive subscale scores were not substantially different (*p* = 0.367). In the general linear model repeated measures, the time‐treatment interaction had no statistically significant impact on the PANSS‐positive subscale scores [*F* (2.291, 164.98) = 0.511, *p* = 0.625, η^2^ = 0.007] (Figure 2B). At any time point, there was no significant difference in PANSS‐positive subscale scores between the two groups (Table 2).

#### 3.1.3 PANSS general psychopathology subscale

When the two groups' baseline PANSS general psychopathology subscale scores were compared, there was no significant difference (*p* = 0.888). The PANSS general psychopathology subscale scores significantly changed as a result of the time‐treatment interaction in the general linear model repeated measures [*F* (2.828, 203.59) = 28.826, *p* < 0.001, η^2^ = 0.286] (Figure 2C). After six and 8 weeks of treatment, the pentoxifylline group demonstrated a statistically significant drop in PANSS general psychopathology subscale scores as compared to the placebo group (Table 2).

#### 3.1.4 PANSS total score

When the two groups' baseline PANSS total scores were compared, there was no significant difference (*p* = 0.444). The PANSS total scores significantly changed as a result of the time‐treatment interaction in the general linear model repeated measures [*F* (2.533, 183.347) = 66.56, *p* < 0.001, η^2^ = 0.48] (Figure 2D). After six and 8 weeks of treatment, the pentoxifylline group had a statistically significant drop in PANSS total scores as compared to the placebo group (Table 2).

#### 3.1.5 Hamilton depression rating scale

The baseline HDRS total score in the pentoxifylline group was 7.35 ± 0.95, whereas in the placebo group it was 7.55 ± 0.85, with no statistically significant difference between the two groups (*p* = 0.323). After treatment, HDRS total score in pentoxifylline group was 7.43 ± 0.8, whereas in the placebo group was 7.71 ± 0.8 with no statistically significant difference between the two groups (*p* = 0.131).

#### 3.1.6 Extrapyramidal symptoms rating scale

The baseline ESRS total score in pentoxifylline group was 1.78 ± 0.42 and 1.73 ± 0.45 in the placebo group, with no statistically significant difference between the two groups (*p* = 0.606). In the general linear model repeated measurements, the time‐treatment interaction had no statistically significant impact on the ESRS scores [*F* (2.886, 207.5) = 0.661, *p* = 0.571, η^2^ = 0.009]. After treatment, ESRS total score was 1.7 ± 0.46 in pentoxifylline group and 1.81 ± 0.4 in the placebo group, with no statistically significant difference between the two groups (*p* = 0.285).

### 3.2 Effect on cAMP and selected inflammatory cytokines

There was no statistically significant difference in baseline cAMP, TNF‐α, and IL‐6 serum levels between the pentoxifylline and placebo groups. (*p* > 0.05). After 8 weeks of treatment, the pentoxifylline group had statistically significant increases in cAMP serum levels as compared to the placebo group (*p* < 0.001). Contrarily, when compared to the placebo group, patients who took pentoxifylline had statistically significant lower serum levels of TNF‐α and IL‐6 (*p* < 0.001) as presented in Table 3.

**TABLE 3:** Changes in cAMP and inflammatory markers

Groups	Placebo group (*n* = 37)			Pentoxifylline group (*n* = 37)			*p* value^a^ Baseline	*p* value^a^ Week 8
Parameters	Baseline	Week 8	*p* value^b^	Baseline	Week 8	*p* value^b^		
cAMP (ng/ml)	30.7 ± 5.59	31.48 ± 5.55	0.135	29.45 ± 4.26	52.64 ± 8.33	<0.001	0.285	<0.001
TNF‐α (pg/ml)	27.87 ± 4.37	26.73 ± 4.76	0.149	26.86 ± 4.36	13.54 ± 3.26	<0.001	0.318	<0.001
IL‐6 (Pg/ml)	44.2 ± 11.12	43.15 ± 10.45	0.165	44.66 ± 10.67	24.39 ± 4.04	<0.001	0.860	<0.001

*Note*: Data presented as mean ± SD. cAMP, cyclic adenosine monophosphate; IL‐6, Interleukin 6; TNF‐α, tumor necrosis factor alpha.

^a^ Baseline and 8‐week comparisons between groups.

^b^ Within group comparison.

Furthermore, cAMP serum level in the pentoxifylline group was significantly higher after 8 weeks compared with their baseline data (*p* < 0.001). Moreover, TNF‐α and IL‐6 serum levels in the pentoxifylline group were statistically significant lower after 8 weeks compared with their baseline data (*p* < 0.001). Contrarily, as compared to the baseline data, the cAMP, TNF‐α, and IL‐6 serum levels in the placebo group after 8 weeks of treatment were not significantly different (*p* = 0.315), (*p* = 0.149), and (*p* = 0.165), respectively.

Notably, the pentoxifylline group's PANSS‐negative subscale scores and cAMP serum levels revealed a statistically significant negative correlation (*r* ^2^ = −0.748, *p* < 0.001), but TNF‐α and IL‐6 serum levels showed a statistically significant positive correlation (*r* ^2^ = 0.743, *p* < 0.001; *r* ^2^ = 0.704, *p* < 0.001).

### 3.3 Clinical side effects

The frequency of side effects was not substantially different between the two groups. In pentoxifylline group, five patients suffered from headache, three from dizziness, five from insomnia, six from abdominal pain, five from heartburn, seven from diarrhea, six from decrease appetite, two from increase appetite, and five from sexual dysfunction. In placebo group, four patients suffered from headache, three from dizziness, four from insomnia, seven from abdominal pain, four from heartburn, six from diarrhea, five from decrease appetite, three from increase appetite, and four from sexual dysfunction. In both groups, no extrapyramidal symptoms were reported.

## 4 DISCUSSION

As far as we know, our study is the first randomized, double‐blind, placebo‐controlled trial that assessing the efficacy and safety of pentoxifylline as PDE inhibitor in alleviating the negative symptoms in chronic schizophrenia. Patients received pentoxifylline showed significant enhancement in PANSS negative, general psychopathology, and total subscale scores relatively to placebo group, but regarding the PANSS positive, the results were non‐significant. Our results could be clinically significant since negative symptoms are principal predictors for further functional impairment in patients suffering from schizophrenia and the current antipsychotics alone do not satisfactorily alleviate these symptoms.^2^ Primary negative symptoms that are associated with schizophrenia are difficult to be assessed because they might be influenced by other aspects such as positive symptoms, overall psychopathological, and other depression‐associated symptoms.^39^ As a result, patients were appropriately stabilized at the beginning of the trial to reduce the impact of these disturbing influences. Furthermore, general linear regression demonstrated that the pentoxifylline group showed significant outcomes in terms of improvement in negative symptoms after correcting for PANSS positive and general, ESRS, and HDRS scores.

A Previous report proved that PDEs are highly expressed in the brain particularly in the striatum, hippocampus, caudate‐putamen, and cortex, which are known to be involved in neuropsychiatric diseases including cognitive dysfunction and negative symptoms in schizophrenia.^18^ Pentoxifylline is a nonselective PDE inhibitor.^32^ Our results showed that pentoxifylline adjuvant therapy led to a substantial increase in the level of cAMP, which could support the survival of dopamine‐secreting neurons. It was reported that the upregulation of cAMP/PKA signaling triggers the synthesis of dopamine at dopaminergic synapse, blocks the dopamine D2‐receptor, and activates dopamine D1‐receptor in striatonigral neurons.^20^, ^21^ In line with our results, it was suggested that rolipram‐induced inhibition of PDE4 upturns the intracellular cAMP in striatum and frontal cortex. Such changes enhance the synthesis and the fate of dopamine in striatum and augment signaling of the dopamine D1‐receptor in frontal cortex.^40^ Similarly, roflumilast, which is also a PDE4 inhibitor, is nowadays a treatment for chronic obstructive pulmonary disease and was suggested as a cognitive enhancer in schizophrenia through enhancing the amplitude of mismatch negativity, working memory‐related theta oscillations, and verbal memory with normalization deficits in attentional set‐shifting and learning‐related activity impairments by increasing intracellular cAMP in brain areas implicated in cognitive deficits in patients with schizophrenia.^41^, ^42^, ^43^ Moreover, our findings were in agreement with a former study reported that cilostazol, PDE3 inhibitor, has improved the negative symptoms in schizophrenia patients in an 8‐week treatment study as an adjunct to risperidone.^44^ Furthermore, inhibition of PDE1 by DSR‐141562 in an animal model exhibits potent efficacy for positive, negative, and cognitive symptoms associated with schizophrenia via augmentation of D1 receptor signaling.^45^

Additionally, the pentoxifylline group's improvement may be attributed to the drug's anti‐inflammatory properties, which led to a significant drop in TNF‐α, and IL‐6 serum levels compared to baseline and patients taking a placebo. Pentoxifylline can also inhibit the production of cytokines and other biomolecules that are responsible for inflammatory cascade, decrease the neutrophil to lymphocyte ratio and thereby reinstating regulatory T cells/T helper‐17 (Treg/Th17) lymphocytes.^46^, ^47^ Moreover, it was suggested that pentoxifylline blocks the neurological deficit score and cerebral infarct volume in cerebral ischemia reperfusion‐induced injury in rats, which was suggested to be mediated through the anti‐inflammatory, antioxidant, and antiapoptotic mechanisms.^48^ Patients with deficits have been found to have higher levels of proinflammatory cytokines such TNF‐α and IL‐6 compared to both nondeficit patients and healthy controls.^49^ In addition, these cytokines may interfere with 5‐hydroxytryptamine (5‐HT) synthesis and glutamatergic transmission through reducing the action of indoleamine 2,3‐dioxygenase with consequent kynurenic acid accumulation; the endogenous glutamate *N*‐methyl‐D‐aspartate receptor antagonist that is deeply implicated in schizophrenia pathophysiology.^50^, ^51^ Furthermore, it was reported that many antipsychotics can act as indirect immunomodulators, supporting the notion of the participation of immune response in the pathogenesis of schizophrenia.^52^, ^53^

The inflammatory activation of astrocytes can increase kynurenic acid production that results in a decrease in the levels of dopamine, acetylcholine, gamma‐aminobutyric acid, and glutamate.^54^, ^55^, ^56^, ^57^, ^58^ Pentoxifylline suppresses TNF‐α and serum‐induced astrocyte proliferation and signaling via the mammalian target of rapamycin and glial cell cAMP‐elevating action.^59^ In addition, medications causing cAMP elevation were found to increase the production and/or the release of numerous neurotransmitters including glutamate and dopamine.^19^, ^20^ In accordance with these findings, several trials using anti‐inflammatory drugs as an adjuvant to antipsychotic treatments revealed promising outcomes concerning both positive and general symptom scores on the PANSS such as celecoxib, which was also found to have a significant positive effect on major depression.^10^, ^11^ Furthermore, our findings were consistent with the findings of an 8‐week trial of pioglitazone augmentation therapy with risperidone, which demonstrated an enhancement in negative symptoms in patients suffering from chronic schizophrenia and that was attributed to its anti‐inflammatory and antioxidant properties.^9^

Although these encouraging outcomes of our study regarding the safety and efficacy of pentoxifylline in management of negative symptoms of schizophrenia, it had some limitations. We had no guide to make an unambiguous conclusion about the best dosage because this was the first clinical research of pentoxifylline in patients with schizophrenia. Furthermore, the small sample size and the short duration are considered probable limitations of this study. Even yet, PANSS is the “gold standard measure of treatment efficacy” since it offers objective evaluation of clinical response to pharmacological therapy. It still has the flaw of not specifically covering all deficit syndrome, cognitive function, and negative symptom domains.^60^ As a result, future research with large sample sizes and longer period could be able to confirm the efficacy of pentoxifylline in patients suffering from schizophrenia, determining its optimum dose, and exploring further targets by neuroimaging.

## 5 CONCLUSION

Pentoxifylline adjuvant to risperidone enhanced the negative symptoms in chronic schizophrenia patients without remarkable side effects. These effects could be attributed to inhibition of PDEs and inflammatory cytokines. Our findings could indirectly support the role of PDEs and inflammation in the schizophrenia‐negative symptoms pathophysiology. Nevertheless, further trials with larger scale and longer durations are recommended to test the long‐term safety, effectiveness, and optimum dose of pentoxifylline.

## CONFLICT OF INTEREST

The authors state they have no competing or financial interests.

## Data Availability

On reasonable request, the corresponding author will provide the data that underpin the study's conclusions.
